# Cyclic AMP-Response Element Regulated Cell Cycle Arrests in Cancer Cells

This article has been retracted.

**DOI:** 10.1371/journal.pone.0065661

**Published:** 2013-06-28

**Authors:** Ping Wang, Shuaishuai Huang, Feng Wang, Yu Ren, Michael Hehir, Xue Wang, Jie Cai

**Affiliations:** 1 Zhejiang Provincial Key Laboratory of Pathophysiology, Medical School, Ningbo University, Ningbo, China; 2 Ningbo Medical Center, LiHuiLi Hospital, Medical School, Ningbo University, Ningbo, China; 3 Department of Urologic Surgery, Ningbo Urology and Nephrology Hospital, Ningbo University, Ningbo, China; 4 Ningbo Women and Children's Hospital, Medical School, Ningbo University, Ningbo, China; Institute of Molecular and Cell Biology, Biopolis, United States of America

## Abstract

Recently, we have demonstrated that trichosanthin (TCS), a promising agent for the treatment of cervical adenocarcinoma, inhibited HeLa cell proliferation through the PKC/MAPK/CREB signal pathway. Furthermore, TCS down-regulated Bcl-2 expression was abrogated by a decoy oligonucleotide (OGN) to the cyclic AMP-responsive element (CRE). The decoy OGN blocked the binding of CRE-binding protein (CREB) to Bcl-2. These results suggested that CRE-mediated gene expression may play a pivotal role in HeLa cell proliferation. However, little is known about the effect of TCS on cell cycle arrests, particularly, whether the genes involved in cell cycle were regulated by CRE. Our present study shows that the arrests of S, G1 and G2/M phases were accompanied by the significant down-regulation of cyclin A, D1 and CDK 2, 4 in HeLa cells, cyclin D1, E and CDK 2, 4 in Caski and C33a cells, and cyclin A, B1, E and CDK 2 in SW1990 cells. However, the cell cycle arrests were reversed via the significant up-regulation of cyclin A and D1, by the combined treatment of TCS and CRE. In conclusion, these data demonstrate for the first time that specific cell cycle arrests in cancer cells can be induced by TCS by inhibiting the binding of CREB to CRE on genes related to cell proliferation.

## Introduction

Trichosanthin (TCS), an active component isolated from the root tubers of the Chinese medicinal herb *Trichosanthes kirilowii* [1], is a promising agent for the treatment of cancer [2]. Our previous reports showed that TCS inhibited cervical adenocarcinoma HeLa cell proliferation [3] through the PKC/MAPK/CREB signal pathway [4]. Furthermore, TCS down-regulated Bcl-2 expression [5], which was abrogated by a cyclic AMP-responsive element (CRE, TGACGTCA) decoy oligonucleotide (OGN), blocking the CRE-binding protein (CREB) binding site on Bcl-2 [6]. These results suggest that CRE-mediated gene expression may play a pivotal role in HeLa cell proliferation.

However, little is known about the effect of TCS on cell cycle arrest of HeLa cell, cervical squamous carcinoma (Caski and C33a cell), and human pancreatic carcinoma (SW1990 cell), especially, whether genes related to cell cycle were regulated by the CRE decoy OGN.

In the present study, we further explored the effects of TCS on the proliferation of cancer cells, cell cycle arrests in the progress of cell proliferation and the role of CRE in cell cycle regulation.

The aim of this study was to investigate the effects of TCS on cancer cell proliferation and the effect of CRE on TCS-induced cell cycle arrests. An important question was whether CRE-combined cyclins played a critical role in the regulation of cell cycle arrest in these cancer cells.

## Materials and Methods

### Cell lines and culture

Cervical cells (HeLa, Caski, C33a) and SW1990 cells were obtained from American Type Culture Collection (ATCC, USA). HeLa, Caski, C33a [7] and SW1990 cell [8] were grown in monolayer in RPMI 1640 medium (Gibco, NY, USA) and Dulbecco's modified Eagle's medium (DMEM), containing 10% heat-inactivated fetal bovine serum, 100 U/ml of penicillin and 100 µg/ml of streptomycin (BioWhittaker, Inc., Walkersville, MD, USA), in a CO_2_ incubator (Forma Scientific, USA). The medium was replaced twice a week, and cells were passaged every 4–5 days at a ratio of 1∶3.

### Cell treatment

Cells were plated at 2×10^6^ cells/dish in 100-mm dishes in the basal medium. At confluence, they were washed briefly with PBS and then treated with TCS (Jinshan pharmacy company, Shanghai, China). Control cells were incubated in TCS-free medium.

### Cell viability assay

Cell viability was assessed with Cell Counting Kit-8 (Dojindo Laboratories, Kumamoto, Japan) using the methods described previously [3], [4], [9].

### Treatment of cells with CRE-OGNs

CRE decoy OGN (5′-TGACGTCAGAGAGCGCTCTCTGACGTCA-3′) and control OGN (5′- TGACGTCATGACGTCATGACGTCA-3′) were converted to phosphorothioate OGNs (Invitrogen Carlsbad, CA, USA) as previous described [5], [6], [10].

### Preparation of cytosolic and nuclear proteins

The preparations of cytosolic and nuclear proteins were performed as previously described [6], [11], [12]. Briefly, at the end of each designated treatment, cells were washed briefly with cold PBS and lysed by scrapping them in 0.5 ml cold hypotonic buffer (10 mM HEPES, 40 mM KCl, 3 mM MgCl_2_, 1 mM dithiothreitol, 0.2% NP-40, 1 µg/ml aprotinin, 2 µM leupeptin, 1 mM phenylmethylsulfonyl fluoride, 40 mM p-nitrophenyl phosphate, 1 mM sodium orthovanadate and 50% glycerol). The lysates were collected and incubated on ice for 5 min, then centrifuged at 15,000×g for 20 s. The supernatant was collected and saved as the cytosolic fractions. The pellet (i.e. cell nuclei) was resuspended in hypertonic buffer (20 mM HEPES, 420 mM KCl, 1.5 mM MgCl_2_, 0.2 mM EDTA, 0.5 mM dithiothreitol, 0.2% NP-40, 1 µg/ml aprotinin, 2 µM leupeptin, 0.5 mM phenylmethylsulfonyl fluoride, 40 mM p-nitrophenyl phosphate, 1 mM sodium orthovanadate and 25% glycerol). After incubation on ice for 60 min, the samples were centrifuged at 15,000×g for 20 min and the supernatants were collected and saved as nuclear extracts. The cytosolic fractions and nuclear extracts were boiled for 10 min and dissolved in 8% SDS PAGE.

### Cell cycle analysis

For flow cytometry analysis of cell cycle, 1×10^6^ cells were harvested by centrifugation, washed with PBS and fixed with ice-cold 70% ethanol overnight. Fixed cells were treated with 25 µg/ml RNase A at 37°C for 30 min and then stained with propidium iodide (PI) (50 µg/ml, Sigma) solution for 30 min in the dark. The fluorescence intensity of individual cells was measured by a flow cytometer (Beckman Coulter, Inc., Miami, FL, USA). At least 10,000 cells were counted [13].

### Western blot analysis

Total cell lysates were prepared by lysis of cells with radioimmunoprecipitation assay buffer and protein concentration was determined using the protein assay kit (Bio-Rad). For Western blot analysis, 50 µg of each sample was processed as described [14]. The following antibodies were used: anti-cyclin A, B1, D1, E, anti-CDK2, 4 and anti-actin (Cell signaling Thehnology, Inc., Beverly, MA). The secondary antibodies were coupled to horseradish peroxidase and detected by chemiluminescence (Bio-Rad, Hercules, CA). The relative amounts of immunoreactive protein in each band were determined by scanning densitometric analysis of the X-ray films.

### Statistical analysis

All experiments were repeated three times. The data were expressed as means ± SD. ANOVA was used to evaluate the differences between groups. Data reported as mean ± SD of three independent experiments. Differences were considered significant if *p* <0.05.

## Results

### Effects of TCS on the proliferation of cancer cells

TCS of 20–100 µg/ml inhibited the proliferation of cells by 3% to 70% after treatment for 24 h (Fig. 1). The 50% inhibitory concentration (IC_50_) of TCS on Caski and C33a cells was found to be 60 µg/ml, lower than that on HeLa and SW1990 cells (100 µg/ml) (Table 1).

**Figure 1:** Effects of TCS on cancer cell proliferation. TCS inhibited cell proliferation in a dose-dependent manner. Data represent means ± SD of three independent experiments (*p <0.05 compared with control).

**Table 1:** Concentration producing 50% growth inhibition (IC50) of TCS on cancer cells.

Cell line	IC50 (μg/ml)	
	24 h	48 h
HeLa	98.25±1.46	64.21±2.45
Caski	51.46±4.59	22.86±4.63
C33a	49.83±4.21	21.94±2.48
SW1990	101±3.84	73.14±3.51

### Effects of TCS on cell cycle progress and cell cycle regulatory proteins

TCS-treated cancer cells were analyzed by flow cytometry. A dose-dependent cell number increases of S, G1, G2/M phase were shown in HeLa, Caski, and SW1990 cells respectively, after they were treated for 24 hours, (Table 2). The levels of cell cycle related proteins were determined by Western blot assay. TCS decreased the abundance of cyclin A, D1 and CDK 2, 4, while it had no marked effect on the expression of cyclin B1 and E in HeLa cell (Fig. 2). In Caski cell, cyclin D1, E and CDK 2, 4 were significantly decreased, whereas no marked changes were shown in the expression of cyclin A and B1 (Fig. 3). Similar results were found in C33a cells (data not shown). In SW1990 cell, cyclin A, B1, E and CDK 2 were significantly down-regulated, no distinct effects were observed in the expression of cyclin D1 and CDK4 (Fig. 4).

**Figure 2:** Effects of TCS on HeLa cell cycle progress and cell cycle regulatory proteins. HeLa cells were treated with indicated doses of TCS for 24 h. Cell number of S phase increased significantly (A) and expressions of cyclin A, D1 and CDK2, 4 significantly decreased (B). Data represent means ± SD of three independent experiments (*p <0.05 compared with control).

**Figure 3:** Effects of TCS on Caski cell cycle progress and cell cycle regulatory proteins. Caski cells were treated with indicated doses of TCS for 24 h. Cell numbers at G1 phase increased significantly (A) and expressions of cyclin D1, E and CDK2, 4 significantly decreased (B). Data represent means ± SD of three independent experiments (*p <0.05 compared with control).

**Figure 4:** Effects of TCS on SW1990 cell cycle progress and cell cycle regulatory proteins. SW1990 cells were treated with indicated doses of TCS for 24 h. Cell numbers at G2/M phase increased significantly (A), the expressions of cyclin A, B1, E and CDK2 significantly decreased (B). Data represent means ± SD of three independent experiments (*p <0.05 compared with control).

**Table 2:** Cell cycle effects of TCS on cancer cells.*n* = 3, Mean ± SD.

Group	HeLa			Caski			SW1990		
	G1	S	G2/M	G1	S	G2/M	G1	S	G2/M
Control	45.85±2.12	31.79±1.51	22.36±3.04	40.99±1.34	8.97±2.51	50.04±0.38	66.68±3.21	31.12±1.11	2.2±1.24
20 μg/ml	37.23±4.28	44.46±3.19	18.31±0.97	53.42±2.47	2.98±1.18	43.60±1.63	56.15±1.56	23.49±2.0	20.36±1.56
60 μg/ml	26.93±3.47*	49.13±0.42*	23.94±1.15	66.15±2.19*	2.99±0.99	30.86±2.10	35.58±2.41*	21.22±1.54	43.20±1.98*
100 μg/ml	21.12±3.42*	57.85±2.63*	21.03±2.54	80.67±3.44*	1.33±2.61*	18.0±3.51*	11.88±2.54*	22.27±1.57	65.85±1.67*

* *p <0.05 vs* control group.

### Effects of CRE-decoy on the cell cycle progress and regulatory proteins

The arrests of S, G1 and G2/M phases induced by TCS in HeLa (Fig. 5), Caski (Fig. 6) and SW1990 (Fig. 7) cells, were significantly attenuated by the combined treatment of TCS and CRE (A, B). It was found that the TCS-induced decreases of cyclin A and D1 were markedly reversed by the addition of CRE, in HeLa cells (Fig. 5, C, D), Caski cells (Fig. 6 C, D) and SW1990 cells (Fig. 7 C, D).

**Figure 5:** Effects of CRE-decoy on HeLa cell cycle progress and regulatory proteins. TCS-induced increase of cell numbers in S phase was significantly attenuated by the combined treatment of TCS + CRE (A, B). The down-regulated expression of cyclin A and D1 was reversed by TCS + CRE. No effect was observed on other proteins (C, D). Data represent means ± SD of three independent experiments (*p <0.05 compared with control, ^#^ *p* <0.05 compared with TCS).

**Figure 6:** Effects of CRE-decoy on Caski cell cycle progress and regulatory proteins. TCS-induced increase of cell numbers in G1 phase was significantly attenuated by TCS + CRE (A, B). The down-regulated expression of cyclin D1 was reversed by the treatment of TCS + CRE. No effect was observed on other proteins (C, D). Data represent means ± SD of three independent experiments (*p <0.05 compared with control, ^#^ *p* <0.05 compared with TCS).

**Figure 7:** Effects of CRE-decoy on SW1990 cell cycle progress and regulatory proteins. TCS-induced increase of cell number in G2/M phase was significantly attenuated by the treatment of TCS + CRE (A, B). Down-regulated expression of cyclin A was reversed by the treatment of TCS + CRE. There was no effect on other proteins (C, D). Data represent means ± SD of three independent experiments (*p <0.05 compared with control, ^#^ *p* <0.05 compared with TCS).

## Discussion

This study showed, for the first time, that TCS exerted cytotoxic effects on cancer cell viability in a dose-dependent manner (Fig. 1). Caski and C33a cells were sensitive to its inhibitory effect on cell proliferation (Table 1). The results of it's anticancer mechanisms clearly show that the increase of S phase in HeLa cells accompanied the decrease of G_1_ phase cells, while the number of G_2_ phase cells did not change. In Caski and C33a cells, significant increase of G_1_ phase and decrease of S and G_2_ phase cells were observed. In SW1990 cells, an increase of G_2_/M phase cells was accompanied by a decrease of G_1_ phase cells, with no change found in the number of S phase cells (Table 2).

Investigating the changes in multiple regulatory molecules involved in the cell cycle showed that the expressions of cyclin A, D1 and CDK 2, 4 in HeLa cells (Fig. 2), cyclin D1, E and CDK 2, 4 in Caski and C33a cells (Fig. 3), cyclin A, B1, E and CDK 2 in SW1990 cells (Fig. 4) were significantly down-regulated. Blocking the binding site of cell cycle genes to CREB by OGN, a CRE decoy, prevented the TCS-arrested S, G1 and G2/M cell cycles in HeLa (Fig. 5 A, B), Caski (Fig. 6 A, B) and SW1990 (Fig. 7 A, B) cells, respectively. The TCS mediated down-regulation of cyclin A, D1 in HeLa cells (Fig. 5 C, D), cyclin D1 in Caski cells (Fig. 6 C, D) and cyclin A in SW1990 cells (Fig. 7 C, D) were reversed by the combination of CRE and TCS.

These results confirmed and extended our earlier reports showing that TCS has a cytotoxic effect on cancer cells [3], [4], and partly revealed the mechanisms underlying the activation of CREB protein [5], [6]. However, it has not been previously reported whether TCS-mediated cell cycle arrest occurs through the combination of CRE and target genes. The present study shows that CRE decoy OGN attenuated the decrease of the expressions of cyclin A and D1 resulting from TCS treatment, and reversed the cell cycle arrests.

The cell cycle is tightly mediated through a complex network of positive and negative cell-cycle regulatory molecules such as CDKs, CKIs and cyclins [15], [16]. It has been reported that the formation of active cyclin D/CDK4 and cyclin E/CDK2 complexes controls the progression through G1 phase (G1/S transition). Further, cyclin A binds to and activates CDK2, promoting G1/S and G2/M cell cycle transitions. In late G2, cyclin B/CDK2 is activated, allowing entry into mitosis [17]. In the present study, we found that the decreased expressions of cyclin A, D1 and CDK2, 4 were associated the S phase arrest in HeLa cells (Fig. 2). The decreased-expressions of cyclin D, E and CDK2, 4 were related to G1 phase in Caski and C33a cells (Fig. 3). The expressions of cyclin A, B1 and CDK2 were significantly down-regulated in SW1990 cells, arrested in G2/M phase (Fig. 4). We also found that CDK2 was significantly decreased in cell lines. This result accords with the notion that CDK2 has a distinct and essential function in the mammalian cell-cycle, and its mutation or inhibition causes a G1-phase block [18].

The activation of genes bearing CRE is reported to occur by phosphorylating CREB at Ser 133 and binding to CRE consensus sequences in the promoter region of genes [19], [20]. CREB phosphorylation peaks during the G1-S transition and then gradually decreases from S phase to M phase [21]. Combined with our previously reported results [4]–[6], [9], it is logical to hypothesize that cell proliferation genes, bearing the CRE site, bind to CREB and affect its phosphorylation level, thereby interfering with cell division.

CRE locates upstream of the mRNA start sites. It has a key role in the cyclin A [22], [23] and D1 [24], [25] expression via CREB activation [26]–[28]. A previous study showed that the association of CREB with vaccinia-related kinase 1 (VRK1) occurred in a cell-cycle-dependent manner from late G1 to S phase. Furthermore, VRK1 specifically enhanced the activity of CRE in cyclin D1 promoter by facilitating the recruitment of phosphorylated CREB to this locus [29]. Giampuzzi et al also found that a significant diminution of CREB protein binding to the cyclin D1 promoter led to a dramatic inhibition of cyclin D1 protein expression in lysyl oxidase (LOX)-up-regulated cells [30]. This phenomenon was also confirmed in fibroblast cells [31], endometrial cell [32], INS cell [33], hepatocyte cell [34] and other cell lines [21], [35], [36]. In addition, a number of observations suggested cyclin A plays a pivotal role on S and G2/M transition in mammalian cells and this role is consistent with its preferential association with CDK2, instead of CDC2, during S phase [37], [38]. CRE was confirmed to be required for efficient activation of the cyclin A promoter in aortic smooth muscle cells [39], fibroblast cells [40] and human embryonal carcinoma cells [22]. The present study clearly shows that combined treatment of TCS and CRE attenuated the decreases of cyclin A and D1 expression, thereby reversing the effect of TCS on cell cycle arrest. Therefore, we suggest that transcription factor CREB is one of the upstream regulators of TCS-induced cell cycle arrest in cancer cells.

## Conclusion

Our findings show, for the first time, that TCS induces specific cell cycle arrests in cancer cells by inhibiting the binding of CREB to CRE on genes related to cell proliferation.
